# Clinical Efficacy and Safety of “Three-Dimensional Balanced Manipulation” in the Treatment of Cervical Spondylotic Radiculopathy by Finite Element Analysis

This article has been retracted.

**DOI:** 10.1155/2021/5563296

**Published:** 2021-03-31

**Authors:** Shengnan Cao, Yuanzhen Chen, Feng Zhang, Shifei Sun, Congan Wang, Guangjian Hou, Dandan Wang, Guodong Sun, Bin Shi

**Affiliations:** ^1^School of Acupuncture-Tuina, Shandong University of Traditional Chinese Medicine, Jinan 250014, China; ^2^Bone Biomechanics Engineering Laboratory of Shandong Province, Neck-Shoulder and Lumbocrural Pain Hospital of Shandong First Medical University, Jinan 250062, China; ^3^School of Precision Instrument and Optoelectronics Engineering, Institute of Medical Engineering and Translational Medicine, Tianjin University, Tianjin 300072, China; ^4^Department of Rehabilitation Medicine, The Third Affiliated Hospital of Shandong First Medical University, Jinan 250031, China

## Abstract

Cervical spondylotic radiculopathy (CSR) is the most commonly encountered cervical spine disorder. Cervical manipulation has been demonstrated as an effective therapy for patients. However, the mechanisms of manipulations have not been elucidated. A total of 120 cervical spondylotic radiculopathy patients were divided into the “three-dimensional balanced manipulation” treatment group (TBM group) and control group randomly. The control group was treated with traditional massage; the TBM treatment group was treated with “three-dimensional balanced manipulation” based on traditional massage. The symptoms and clinical efficacy of the patients were compared before and after treatment for one month. A three-dimensional finite element model was established. The mechanical parameters were imported to simulate TBM, and finite element analysis was performed. The results showed that the total effective rate was significantly higher in the TBM group compared with the control group. The biomechanical analysis showed the vertebral body stress was mainly distributed in the C3/4 spinous processes; the deformation mainly concentrated in the anterior processes of the C3 vertebral body. The intervertebral disc stress in the C3~C7 segment was mainly distributed in the anterior part of the C3/4 intervertebral disc, and the deformation extends to the posterior part of the C3/4 nucleus pulposus. In summary, these data are suggesting that TBM was effective in CSR treatment. The results of the finite element model and biomechanical analysis provide an important foundation for effectively avoiding iatrogenic injuries and improving the effect of TBM in the treatment of CSR patients.

## 1. Introduction

Cervical spondylotic radiculopathy (CSR) is the most commonly encountered cervical spine disorder among middle-aged and elderly people, accounting for 60% to 70% of cervical spondylosis cases in China [1]. Conservative therapy and surgical interventions are the most common treatment strategies for CSR. Manipulation therapy is considered an efficacious and cost-effective approach for the management of CSR [2], which has the effect of releasing adhesions, relieving muscle spasms, and correcting the joint dislocation in the treatment of CSR and has been widely used in the clinic for treating CSR patients [3]. Based on traditional rotatory manipulation and comprehensive consideration of cervical anatomy, physiology, and biomechanics, we developed a manipulation therapy named “three-dimensional balanced manipulation” (TBM) and widely used this TBM in the treatment of CSR patients [4]. The most prominent feature of TBM is to decompose the core operations of rotary thrust into a fixed rotary position, the forward thrust of the operator, the instantaneous rotational force, and the upward thrust of the operator.

During the treatment of manipulation, the stress distribution in different parts of the cervical spine is critical to the safety of the manipulation. If the stress exceeds the normal range, the manipulation may damage the articular process joints, resulting in excessive protrusion of the intervertebral disc. However, the biomechanical mechanism of manipulation therapy for the treatment of conditions involving the cervical vertebra has not yet been elucidated. This is because that there is a scarcity of specimens for in vitro investigations and the distribution of and changes in stress within the cervical vertebrae cannot be measured by traditional experimental methods [5]. Therefore, a new detection method is urgently needed.

Finite element analysis (FEA) has been used to investigate the biomechanics of the cervical spine [6, 7]. It can provide information about stress distribution, deformation, and strain on any part of the cervical vertebrae during simulated manipulations, containing flexion, extension, and torsion [8]. Recently, different finite element models (FEM) of the cervical spine were constructed to investigate the biomechanics of the cervical spine or intervertebral disc [9–11]. However, few studies have established a FEM based on CSR, and few studies have performed biomechanical analysis of stress distribution, deformation of the model when imitating manipulation therapy.

This study was aimed to determine the effectiveness of TBM on CSR, and FEA was used to study the stress distribution and changes in the cervical spine during TBM treatment to investigate the safety and effectiveness of the TBM. The results will provide important support for the clinical efficacy and safety of TBM in the treatment of CSR.

## 2. Methods

### 2.1. CSR Patients

This study was officially approved by the Ethics Committee of Shandong Academy of Medical Sciences. Written consent was obtained from each patient for participation in the study. A total of 122 CSR patients were selected from January 2019 to March 2020 from the Neck-Shoulder and Lumbocrural Pain Hospital of Shandong First Medical University. The patients were divided into the TBM treatment and control groups by using the random number table method according to the order of treatment.

### 2.2. Treatment

The control group was treated with traditional massage, and the TBM treatment group was treated with TBM based on traditional massage. Manipulative treatment included adjustment of the left and right sides.

TBM treatment: consider a C4/5 left lesion and the C5 spinous process with a relatively left displacement as an example. The patient was in a sitting position. An assistant physician fixed the patient's lower limbs. The doctor held the left thumb to the right side of the C5 spinous process, and the other four fingers reached the occiput. The patient was advised to relax, the neck flexing 10°~20° with the jaw placed on the right elbow of the doctor. The doctor slowly pulled the patient's neck with light force for about 1~2 min and, then, slowly rotated the patient's head and neck to the right until a resistance was encountered. At this point, the doctor forced the patient's head and neck to the right side with the right elbow and pushed the C5 spinous process to the left with the left thumb, with a reset of C5 spinous process or an audible cracking sound during manipulation. The same manipulation was used to reverse adjust the C4 spinous process. The patient placed on the back for clinical observation for 20 min. The patient received TBM treatment once every other day and 10 treatments constituted a course and follow-up after 1 month.

Traditional massage: the patient was in a sitting position. The doctor pressed and kneaded the patient's acupoints of Tianzong (SI11), Dazhui (GV14), Fengfu (GV16), and Fengchi (GB20), with his/her thumb, each for 5 min. Massage therapy was performed once every other day, and 10 treatments constituted a course, and follow up after 1 month.

### 2.3. Efficacy Evaluation

Clinical efficacy was evaluated based on the Visual Analogue Scale (VAS) and clinical efficacy standard against CSR according to “Diagnostic and Efficacy Criteria for TCM Disorders” promulgated by National Chinese Medicine in 1994.

Visual Analogue Scale (VAS): the VAS table was supervised by the Chinese Medical Association Pain Society. Patients marked the points on the back of the ruler according to their sense of pain. The VAS score was determined by the centimeters from the left end of the ruler to the point marked by the patient. VAS scores ranging from 0 to 10 were defined as follows: 0 (indicated a lack of pain, 0 cm), 1~3 (mild pain and do not affect work and life, 1~3 cm), 4~6 (moderate pain affecting work but not life, 4~6 cm), and 7~10 (severe pain affecting work and life, 7~10 cm).

Evaluation of clinical efficacy: the condition was considered to have been cured if the original discomfort disappeared, normal muscle strength was gained, the function of the neck and affected limbs recovered, and if the patient could participate in laborious activities and work normally. The patient was considered to show an improvement if the original symptoms obviously resolved, neck and shoulder pain disappeared, and limb function obviously improved. The treatment was considered ineffective if the symptoms and signs did not show any improvement. The calculation of cure rate: cure number/total number × 100%; the calculation of total efficiency rate: (cure number + improvement number)/total number × 100%.

### 2.4. C3~C7 FEM Establish and Loading Conditions

FEM was reconstructed based on axial Computed Tomography (CT) images of a 39-year-old male CSR patient; the data were recorded and stored in the Digital Imaging and Communications in Medicine (DICOM) format. A three-dimensional FE model of the C3~C7 segments of the CSR was extracted and established using the Mimics 20.0 (Materialise, Inc., Leuven, Belgium) software. The model was further optimized using tools such as Grid Editing in the Geomagic Studio 2015 (Raindrop Geomagic, Inc., Morrisville, NC) software to obtain a high-quality, curved, smooth solid model similar to the cervical vertebrae of patients with actual radiculopathy. The abovesaved entity model was imported into the ANSYS Workbench 18.1 (ANSYS, Inc. Pennsylvania, America) software, and the ligament was created by the geometry concept modeling function. The ligament start and end points and cross-sectional area were determined according to published literature [12–15]. The cervical vertebrae consisting of cortical and cancellous bones were simulated using Solid187 solid element. The CPT217 void pressure unit was used to simulate the intervertebral disc (nucleus pulposus and annulus fibrosus). The five ligaments were simulated by a nonlinear spring and connected to the relevant nodes. The facet joint was considered to be a nonlinear three-dimensional contact, modeled by a face-to-surface contact element with a coefficient of friction of 0.1. The mechanical properties of the isotropic elastic biomaterials in this study were assumed to be homogeneous and continuous. When force was applied, the cut surfaces of the model did not slide against each other, and each unit had sufficient stability.

The boundary conditions and loading conditions were set as follows: constrained the lower surface of the C7 vertebral body, and all nodes on the lower surface were completely fixed. The uppermost C3 was free from any constraints and accepted the load vector. A compressive load was applied to the superior part of the model to represent the head weight. Other types of loading, including tension, compression, lateral bending, and axial rotation, can be applied on the superior part of the uppermost vertebra body. To validate the movement and flexibility of the model, by setting the boundary and loading conditions, the flexion and extension, and rotation of the cervical spine in physiological conditions were simulated, and the motion angle were recorded and compared with the research results [10] to verify the mobility of the C3~C7 three-dimensional FEM.

### 2.5. Simulation of TBM

Consider a C4/5 left lesion and the C5 spinous process with a relative left displacement as an example. The present study simulated the left lateral lesion of C4/5 and TBM of the C5 spinous process with a relatively left displacement. For TBM in the sitting position, the patient sat upright, and the bottom of the C7 vertebral body and the joint surface of the inferior articular process were fixed with fixed support constraint. A 5 kg downward force was applied to the upper surface of the C3 vertebral body. Then, TBM was slightly lifted and vertical traction force of 4.2 kg was applied to the top of the C3 vertebral body. The C5 spinous process was slowly rotated with 20° flexion and 1.0 N.m torque.

### 2.6. Statistical Analysis

Statistical analyses were performed with the Statistical Package for the Social Sciences, version 24.0 (SPSS Inc., Chicago, IL, USA). Clinical efficacy was analyzed using the *χ*^2^ test. The two-tailed unpaired Student's *t*-test was used to assess differences in VAS between different groups. A paired *t*-test was used to analyze intragroup differences. All data were described as mean ± standard deviation ($\bar{x}\pm S$) values, and a two-sided *P* value of less than 0.05 considered to be statistically significant.

## 3. Results

### 3.1. The Efficacy of TBM in the Treatment of CSR Patients

In a comparison of the changes in symptoms and signs before and after treatment in the control and TBM groups, the VAS scores in the two groups were obtained before treatment (*P* > 0.05). After one course of treatment, the VAS scores in the two groups after treatment were significantly lower than those before treatment (*P* < 0.01), and the VAS score in the TBM group was significantly lower than that in the control group (*P* < 0.01, Figure 1(a)) after treatment. The findings of clinical evaluation of CSR patients were statistically analyzed. The cure rate in the TBM group was significantly higher than that in the control group (50.00% and 33.33%, respectively, *P* < 0.05). The total effectiveness rate in the TBM group was significantly higher than that in the control group (95.00% vs. 76.67%, *P* < 0.05, Figure 1(b)).

### 3.2. Stress Distribution of the C3 ~ C7 Vertebral Body

The TBM in the sitting position was decomposed and simulated. When the model was loaded with a downward force of head gravity, the stress was mainly concentrated at the vertebral body and the articular process (Figure 2(a)). As the upward traction increased, the stress was mainly concentrated at the C4 spinous process and articular process, C5 vertebral arch, spinous process and articular process, C7 transverse process, and articular process (Figure 2(b)). When a 1.0-N.m rotating torque of 20° left anterior was loaded on the model, the stress distribution of the C5 spinous process gradually increased and extended to the posterior part of the spinous process and the vertebral arch. When the combined force reached the maximum level, the stress on the C3~C7 vertebral body reached the maximum value of 17.781 MPa. Stress was concentrated at the C3~C4 spinous processes, anterior region of the C5 spinous process, spinous process root, vertebral arch, and the combination of the C6~C7 joints (Figure 2(c)).

Deformation of the vertebral body corresponded to the stress distribution. When the model was loaded with a downward force of head gravity, the vertebral deformation showed that the maximum displacement was located at the front end of the C3 vertebral body and the transverse process and was gradually distributed around the posterior vertebral body, the vertebral arch, and the superior articular process (Figure 2(d)). As the upward traction increased, the model was in tension and the displacement was gradually reduced. The maximum displacement of the whole model was located at the front of the C3 transverse process and the upper articular process (Figure 2(e)). When the model was loaded with a rotating torque of 20° left anterior, the C3 to C7 segments also showed a rotation displacement. The displacement of the model was mainly concentrated at the C3~C4 segments, and the maximum displacement was located at the front of the articular process and transverse process of C3. In addition, the superior articular process and transverse process of C4 and the C5 superior articular process showed slight displacement (Figure 2(f)).

### 3.3. Biomechanical Analysis of Intervertebral Disc of C3~C7

When the model was loaded with a downward force of head gravity, the compressive stress mainly accumulated around the periphery of the nucleus pulposus (Figure 3(a)). When an upward traction was applied to the model, the C3 vertebral body was gradually pulled upward, and the tensile stress was mainly concentrated at the C4/5, C5/6 intervertebral disc (Figure 3(b)). When the rotational torque was loaded on the model, the changes in compressive stress were mainly concentrated at the nucleus pulposus of C4/5 with a value of 30.429 MPa, the anterior disc of C3/4, the nucleus of C5/6, and the posterior part of the C6/7 disc (Figure 3(c)).

Deformation analysis of the intervertebral discs showed that the compression displacement was mainly at the front end of the C3/4 intervertebral disc and the anterior half of the nucleus pulposus with a decreasing distribution to the posterior half (Figure 3(d)). As upward traction was applied to the C3 vertebral body, and the displacement decreased gradually as the tension increased. The stress was concentrated mainly at the anterior part of the annulus fibrosus and nucleus pulposus (Figure 3(e)). With a 1.0-N.m rotational torque loaded on the model, the displacement of the four intervertebral discs increased, and the displacement of the C3/4 intervertebral disc was the largest. The displacement extended to the middle and posterior parts of the C3/4 nucleus pulposus. The displacement of the nucleus pulposus and the anterior disc of the C4/5, C5/6 gradually expanded (Figure 3(f)).

## 4. Discussion

Currently, in the absence of myelopathy or obvious muscle weakness, patients with cervical radicular pain should be treated conservatively [16]. Complementary and alternative medicine interventions for CSR patients have shown a tendency to improve the associated symptoms and clinical signs [17]. Neck pain may be caused by the compression of the lesser and greater occipital nerves by posterior cervical muscles and their fascial attachments at the occipital ridge with subsequent local perineural inflammation. Traditional Chinese manipulation therapy is a frequently applied complementary and alternative medicine intervention to relieve the symptoms of CSR due to its immediate effects on pain and the absence of toxic and side effects [18].

A previous study proposed a TBM based on the traditional rotatory manipulation with comprehensive consideration of cervical anatomy, physiology, and biomechanics [19]. Another study revealed that TBM can relieve muscle spasm, adjusting the relationship between abnormal spine and bone, correcting spinal dislocation, and restoring the biomechanical balance of the spine [20]. In the present study, the clinical efficacy analysis of 120 CSR patients revealed that the cure rate and total effectiveness rate in the TBM group were significantly higher than those in the control group. None of the patients showed adverse reactions during treatment. In the study by Yang et al., the therapeutic effectiveness and safety of balance chiropractic therapy for CSR were investigated [17, 21]. These studies, together with ours, suggest that manipulation therapy has become a widely applied conservative intervention to relieve the symptoms of CSR.

In the present study, despite the widespread use of TBM in clinical practice, little is known about the biomechanical characteristics of TBM. Therefore, the FE analysis was used as a noninvasive approach to investigate stress distribution and displacement in CSR during simulated TBM, which has seldom been reported. Findings from our study would impart useful insight for the spinal manipulators and help to further understand the clinical efficacy of TBM.

A traditional viewpoint holds that decreasing of intradiscal pressure is thought to be helpful for prolapsed discs reabsorption, and intradiscal pressure can be reduced through spinal manipulation [21]. This opinion indicates that spinal manipulation, or TBM, might play a role in reducing intradiscal pressure for treating CSR. In the present study, when the manipulative force was completely loaded on the model, the deformation and displacement extended to the middle and posterior parts of the C3/4 nucleus pulposus, the periphery of the nucleus pulposus of C4/5 and C5/6, and the anterior part of the cervical disc. Since we found that TBM could increase vertebral body and intervertebral disc displacement in a FEM, which may be beneficial for increasing the intervertebral space, expanding the intervertebral foramen, relieving the mechanical compression of the nerve roots by the upper and lower articular processes, and relieving the nerve root compression and stimulating symptoms. This suggested that the clinical efficacy of TBM was associated with the relative displacement between the intervertebral disc and the adjacent nerve root. These mechanisms of clinical efficacy of TBM in the treatment of CSR need to be further investigated in future studies.

When the rotational torque was loaded on the model, the maximum von Mises stress value increased to 17.781 MPa in the anterior region of the C5 spinous process, and the intervertebral disc of C4/5 with a value of 30.429 MPa. It is far less than the initial stress of vertebral fractures [22]. Therefore, the TBM used in the treatment with CSR is within the safe range and will not cause normal cervical vertebrae, pedicles, spinous processes, facet joints, and other bone structural damage. The FEA results provide an important foundation for effectively avoiding iatrogenic injuries of TBM in the treatment of CSR.

The present study has several limitations. Although the experimental analysis approximated the clinical condition, the FEM of this study selected young people and the C4/5 segment. Future studies will expand the sample size for patients of different ages and study the FEA of multisegment and multiage groups.

## 5. Conclusion

The present study found that TBM was effective in the treatment of CSR patients. The FE model and biomechanical analysis of the C3~C7 cervical segment revealed the stress distribution and displacement of each part during TBM treatment. Our results clarify the stress distribution of different parts of the vertebral body and intervertebral disc during the manipulation process, which provide an important foundation for effectively avoiding iatrogenic injuries and improving the clinical efficacy of TBM in the treatment of CSR. Our study provides a new strategy for complementary and alternative medicine treatment of CSR. The findings of our study would further the understanding of the biomechanical characteristics and clinical efficacy of TBM in the treatment of CSR.

## Figures and Tables

**Figure 1:** “Three-dimensional balanced manipulation” was effective in treating cervical spondylotic radiculopathy. (a) Visual Analogue Scale of “three-dimensional balanced manipulation” group and control group before and after treatment. (b) The clinical efficiency and total effective rate in “three-dimensional balanced manipulation” group and control group. ^∗^*P* < 0.05, ^∗∗^*P* < 0.01.

**Figure 2:** Biomechanical analysis of the C3~C7 segment vertebral body in the process of “three-dimensional balanced manipulation.” (a) Stress distribution when the model was only loaded with a downward force of head gravity. (b) Stress distribution during head loading and upward traction. (c) Side view of the stress distribution of the vertebral body during the complete manipulation. (d) The overall model deformation distribution diagram when only the head gravity is loaded. (e) Distribution map of overall deformation when loading head and upward traction. (f) Side view of the distribution of vertebral body deformation under complete manipulation. (a–c) The color represents stress variety, red represents maximum stress, blue represents minimum stress, and from red to blue represents decreasing stress. (d–f) The color represents deformation variety, red represents maximum deformation, blue represents minimum deformation, and from red to blue means represents decreasing deformation.

**Figure 3:** Biomechanical analysis of the intervertebral disc in C3~C7 segments during the process of “three-dimensional balanced manipulation.” (a) Stress distribution when the model was only loaded with a downward force of head gravity. (b) Stress distribution during head loading and upward traction. (c) Side view of the stress distribution of the vertebral body during the complete manipulation. (d) Distribution map of the overall intervertebral disc deformation when only the head gravity is loaded. (e) Distribution of the overall disc deformation when the head is loaded and upward traction. (f) Deformation distribution of intervertebral disc under complete manipulation. (a–c) The color represents stress variety, red represents maximum stress, blue represents minimum stress, and from red to blue represents decreasing stress. (d–f) The color represents deformation variety, red represents maximum deformation, blue represents minimum deformation, and from red to blue represents decreasing deformation.

## Data Availability

The data used to support the findings of this study are available from the corresponding author upon request.
